The article "Stanniocalcin 2 expression predicts poor prognosis of hepatocellular carcinoma" was retracted in 2024. Reasons: duplicated data; duplicate publication; overlap with earlier publications; unreliable results or conclusions.

# Stanniocalcin 2 expression predicts poor prognosis of hepatocellular carcinoma

**DOI:** 10.3892/ol.2014.2520

**Published:** 2014-09-10

**Authors:** ZHEN-HAI ZHANG, YA-GUANG WU, CHENG-KUN QIN, ZHONG-HOU RONG, ZHONG-XUE SU, GUO-ZHE XIAN

**Affiliations:** Department of Hepatobiliary Surgery, Shandong Provincial Hospital Affiliated to Shandong University, Jinan, Shandong 250021, P.R. China

**Keywords:** stanniocalcin 2, hepatocellular carcinoma, prognosis, biomarker

## Abstract

Previous studies have shown that the expression level of stanniocalcin 2 (STC2) is associated with tumor progression. However, to date, the association between STC2 and clinicopathological factors in hepatocellular carcinoma (HCC) has not been investigated. The clinical significance of STC2 was investigated in 30 fresh HCC samples using western blot analysis and in 240 HCC tissues using immunohistochemical analysis. The level of STC2 in cancerous tissue was higher than in the matched non-cancerous tissues. Using immunohistochemistry, the STC2-positive group exhibited a higher incidence of lymph node metastasis and venous invasion compared with the STC2-negative group. Kaplan-Meier survival analysis revealed that the positive expression of STC2 correlated with poor overall survival (OS) and disease-free survival of HCC patients (P<0.01). STC2 expression was observed to be an independent prognostic factor for OS in HCC patients by multivariate analysis (hazard ratio, 2.39; 95% confidence interval, 1.04–5.89; P=0.013). These data suggest that STC2 expression may be a useful indicator of poor prognosis in HCC patients.

## Introduction

Hepatocellular carcinoma (HCC) is one of the most common types of malignant tumor and is the third leading cause of cancer-related mortality worldwide (1). The global distribution of HCC is disproportional, with the highest incidence reported in Asia and Sub-Saharan Africa, particularly in China. HCC patients exhibit an overall 5-year survival rate of only 5% (2). In total, ~70% of patients experience relapse within five years of undergoing surgery and >80% of recurrences are within the remaining liver tissue (3,4). Patients with HCC often exhibit different outcomes, even when identical clinicopathological features are observed; this suggests that the development and rapid progression of HCC involves numerous complex molecular and cellular events. Therefore, in order to develop novel prognostic factors and improve treatment options, the elucidation of the molecular mechanisms involved in tumor progression and identification of the crucial markers that discriminate between the occurrence and the various stages of HCC is imperative (5).

The stanniocalcin 2 (STC2) protein, encoded by the STC2 gene, is a 32-kDa extracellular matrix protein with a signaling peptide; the protein is involved in a number of physiological processes, including bone development, reproduction, wound healing, angiogenesis and modulation of the inflammatory response (6). The majority of the current research is focused on cellular inflammation and carcinogenesis, due to the increasing evidence demonstrating the local actions of STCs (7). Previous studies have reported that various cancers, including renal cell carcinoma (8) and breast cancer (9) have exhibited increased expression of STC2; however, the clinical significance of STC2 in HCC remains to be investigated. Therefore, the current study aimed to explore the STC2 expression levels in HCC tissues and the correlation with prognosis.

## Materials and methods

### Patients and tissue samples

A total of 30 fresh HCC cancerous tissues and paired adjacent non-cancerous tissues were obtained from HCC carcinoma patients, who had undergone hepatectomy in 2012 at the Department of Hepatobiliary Surgery, Shandong Provincial Hospital Affiliated to Shandong University (Jinan, China). The histological diagnosis of HCC was confirmed by two independent pathologists, and these paired tissue samples were utilized for the western blot analysis of STC2 expression. The fresh tissue was surgically removed, immediately frozen and stored in liquid nitrogen. Additionally, paraffin-embedded, paired cancer tissue and adjacent normal tissue samples, which had been obtained from 240 HCC patients at Shandong Provincial Hospital Affiliated to Shandong University between 2005 and 2008, were utilized for the immunohistochemical analysis of STC2 expression.

The follow-up results for the 240 patients enrolled in this study were obtained according to medical records and telephone interviews. Postoperative follow-up was performed on HCC patients every three months during the initial two years, every six months during the third to fifth year, and annually thereafter, for an additional five years or until mortality. Overall survival (OS) was defined as the time from surgery to patient mortality or the last follow-up. Disease-free survival (DFS) was defined as the time from surgery to disease recurrence or metastasis. The study was approved by the Institutional Ethics Board of Shandong Provincial Hospital Affiliated to Shandong University, and informed consent was obtained from all participants.

### Western blot analysis

Western blot analysis was performed to detect the expression of STC2 in the 30 resected HCC specimens. Frozen HCC specimens were ground in liquid nitrogen and harvested. Tissue samples were lysed in RIPA lysis buffer [phosphate-buffered saline (PBS) containing 1% Triton X-100 and 1 nM phenylmethylsulfonyl fluoride] at 4°C for 30 min and subjected to centrifugation at 12,000 × g for 15 min. The protein concentration was quantified using the BCA protein assay (Pierce Biotechnology Inc., Rockford, IL, USA). Equal quantities of protein (50 μg) were loaded and SDS-PAGE was completed on a 12% SDS-PAGE gel, which was then transferred to nitrocellulose membrane. The membrane was incubated for 60 min in PBS containing 0.1% Tween-20 and 5% skimmed milk to block any nonspecific binding. This was followed by incubation at 4°C with monoclonal rabbit anti-human STC2 antibody (1:1000 dilution; Abcam, Cambridge, MA, USA). The membrane was washed three times for 10 min in PBS with 0.1% Tween-20 and subsequently incubated for 1 h with horseradish peroxidase-conjugated bovine monoclonal anti-rabbit (1:5000 dilution) secondary antibody (Boster Biological Technology Ltd., Wuhan, China) at room temperature. The immumoreactive proteins were then detected using ECL substrate (ECL western blotting detection system; Amersham Pharmacia Biotech, Amersham, UK) according to the manufacturer’s instructions. GAPDH was used as an endogenous protein for normalization. The relative intensity of each lane was quantified by scanning densitometry using Quantity One software (Bio-Rad, Hercules, CA, USA).

### Immunohistochemistry (IHC)

Paraffin-embedded HCC or non-cancerous tissues were assessed using immunohistochemical analysis (n=240). The slides were immersed in EDTA (pH 8.0) and boiled for 10 min in a microwave oven for the antigen retrieval. Following three rinses with PBS, the endogenous peroxidase was blocked with 0.3% hydrogen peroxide for 20 min at room temperature. The slides were incubated with the monoclonal mouse anti-rabbit STC2 antibody (1:50 dilution; Abcam, Cambridge, United Kingdom) in a humidified chamber at 4°C overnight. Following additional wash with PBS for three times, the sections were sequentially incubated with horseradish peroxidase-conjugated secondary antibody (Abcam) at 37°C for 30 min and subsequently washed three times with PBS. Finally, diaminobenzidine tetrahydrochloride was used for the signal development and PBS was used as the negative control.

The total STC2 immunostaining scores were calculated as the product of the percentage positivity of the stained tumor cells and the staining intensity (10). The percentage positivity was scored as 0, <5% staining (negative); 1, ≥5 to <25% staining; 2, ≥25to <50% staining; 3, ≥50 to <75% staining; and 4, ≥75% staining. A staining intensity score of 0, no staining; 1, mild; 2, moderate; or 3, strong was allocated. The percentage positivity of cells and staining intensity were determined under double-blind conditions. The STC2 immunostaining score was calculated as the product of the value of the percentage positivity score plus the staining intensity score, ranging from 0 to 12. The STC2 expression level was defined as the following: −, score of 0–3; +, score of 4–6; ++, score of 7–9; and +++, score of ≥10. Based on these STC2 expression levels, the HCC patients were divided into two groups: negative STC2 expression (− and +) and positive STC2 expression (++ and +++).

### Statistical analysis

The SPSS software, version 15.0 (SPSS, Inc., Chicago, IL, USA) was used for statistical analysis. The χ2 test was used to show the differences in categorical variables. Patient survival and the differences in patient survival were determined by the Kaplan-Meier method and the log-rank test, respectively. A Cox regression analysis (proportional hazard model) was performed for the multivariate analyses of prognostic factors. P<0.05 was considered to indicate a statistically significant difference.

## Results

### Upregulation of STC2 in HCC tissues by western blot analysis

Initially, the expression levels of STC2 protein were analyzed using western blot analysis on 30 HCC cancerous tissues and the paired corresponding adjacent non-cancerous tissues. The western blot analysis revealed that STC2 expression was markedly increased in HCC cancerous tissues, compared with the corresponding non-cancerous tissues (P<0.001; Fig. 1).

### STC2 expression correlates with clinicopathological features in HCC

The correlation between STC2 expression and clinicopathological features in HCC was explored using IHC, performed in 240 HCC tissue samples and the paired adjacent normal tissue samples (Fig. 2). Among the tissue samples, 60.83% (146/240) of HCC cancerous specimens exhibited positive expression of STC2. However, STC2 expression was observed to be positive only in 8.75% (21/240) paired adjacent non-cancerous liver specimens. The associations between STC2 expression and the clinicopathological features are shown in Table I. STC2 expression was significantly correlated with serum α-fetoprotein (AFP) levels (P=0.024), recurrence (P=0.011) and metastasis (P=0.025). No statistically significant correlations were identified between the STC2 expression and the remaining clinicopathological features.

### Correlation between STC2 expression and patient survival

The prognostic value of STC2 expression in HCC patients was also evaluated between those with positive and negative expression of STC2. Kaplan-Meier curve analysis indicated that positive expression of STC2 was significantly correlated with poor clinical outcome of HCC patients. HCC patients with positive STC2 expression exhibited significantly shortened OS and DFS, compared with those with negative STC2 expression (Fig. 3). Multivariate analysis was conducted to investigate the impact of the STC2 expression pattern on the clinicopathological features of HCC patients. Univariate analysis indicated that STC2 expression was a significant prognostic factor for OS (Table II). Based on the multivariate analysis, STC2, metastasis and recurrence where independent prognostic factors for OS. Therefore, STC2 expression may be significant in predicting the OS in HCC patients (hazard ratio, 2.39; 95% confidence interval, 1.04–5.89; P=0.013; Table II).

## Discussion

Although the number of novel treatment strategies under development for HCC is currently increasing, including options such as molecular targeted therapy (11), gene therapy (12) and immunotherapy (13), the therapeutic outcomes remain unsatisfactory, and the survival rate of HCC is low (14). Therefore, the identification of new prognostic markers for the prevention and treatment of HCC is an ongoing challenge.

Overexpression of STC2 has been demonstrated to contribute to poor prognosis or recurrence in colorectal (15), gastric (16) and prostate (17) cancer, as well as neuroblastoma (18) and renal cell carcinoma (8). In ER-positive breast cancers, however, STC2 overexpression has been found to indicate a good prognosis (19,20). This variation between reports suggests that the contribution of STC2 to the development of carcinoma is likely to depend on the cancer type.

Elucidating the underlying mechanism of STC2 in HCC is an ongoing challenge. A recent study demonstrated that the proliferative capacity of a gastric cancer cell line was inhibited by treatment with STC2 siRNA. Furthermore, the authors proposed that STC2 may contribute to cancer development and poor prognosis by controlling proliferation in gastric cancer (21). A number of reports have suggested that cells expressing STC2 exhibit resistance to apoptosis. Ito *et al* (22) reported that STC2 expression contributes to antiapoptotic activity and survival of ischemia nerve cells. Furthermore, STC2 was revealed to protect cells from apoptosis in hypoxic ovarian cancer cell lines (23). Conversely, breast cancer cases exhibiting late relapse were observed to overexpress STC2 in the primary and recurrence sites (24). A previous study has demonstrated that STC2 is highly expressed in tumor vascular endothelial cells, and that this overexpression correlates with postoperative recurrences (25). These observations indicate that STC2 expression in cancer samples may contribute to the development of carcinoma through the host vascular endothelial cells, as well as cancer cells.

In the current study, the STC2 protein levels in HCC and tumor-adjacent non-cancerous tissues were evaluated using western blot analysis and IHC. These analyses indicated that STC2 was highly expressed in HCC compared with the corresponding non-cancerous tissues. Furthermore, positive expression of STC2 in HCC was observed to correlate with certain aggressive clinicopathological characteristics, including AFP levels, recurrence and metastasis in the 240 paraffin-embedded paired tissue specimens. The results from the current study also imply that positive STC2 expression was associated with poor prognosis; STC2 positive expression correlated with OS and DFS in the 240 HCC patients. Notably, STC2 was observed to be an independent prognostic factor in these HCC patients.

In summary, the current study reports the differential expression of STC2 in HCC and the possible use of STC2 as a novel prognostic marker in HCC. The present findings demonstrate that the high expression of STC2 in HCC tissue is associated with poor prognosis in HCC patients. Further studies are required to explore and elucidate the underlying mechanisms of STC2 in HCC. STC2 expression may present a useful prognostic marker in HCC patients.

## Figures and Tables

**Figure 1:** Upregulation of STC2 in hepatocellular cancer tissues compared with paired adjacent non-cancerous tissues by western blot analysis. (A) STC2 protein expression in fresh hepatocellular cancer tissues and paired adjacent non-cancerous tissues from five patients. (B) Semi-quantitative analysis of 30 fresh hepatocellular cancer samples and the paired adjacent noncancerous tissues. STC2, stanniocalcin 2, N, non-tumor; T, tumor.

**Figure 2:** Immunohistochemical analysis of STC2 in hepatocellular carcinoma. (A and B) STC2 was observed in the cytoplasm of liver cancer cells and (C and D) was rarely observed in the adjacent non-tumor liver tissue. A and C, magnification, ×100; B and D, magnification, ×400. STC2, stanniocalcin 2.

**Figure 3:** Positive STC2 expression correlates with the poor prognosis of HCC patients. Kaplan-Meier survival analysis for (A) overall survival and (B) recurrence-free survival in 240 hepatocellular carcinoma patients (log-rank test). STC2, stanniocalcin 2.

**Table I:** Correlations of STC2 expression with clinicopathologic features of hepatocellular carcinoma.

		STC2 expression		
			
Clinicopathologic variables	Cases, n	Negative	Positive	P-value^a^
Gender				0.410
Male	198	80	118	
Female	42	14	28	
Age, years				0.390
≤60	191	82	109	
>60	49	12	37	
Liver cirrhosis				0.520
Yes	171	54	117	
No	69	40	29	
Serum AFP, μg/l				0.024
≥400	127	36	91	
<400	113	58	55	
Histological differentiation				0.260
Well	67	31	36	
Moderate	71	11	60	
Poor	102	52	50	
Recurrence				0.007
Present	167	52	115	
Absent	73	42	31	
Metastasis				0.025
Present	162	53	109	
Absent	78	41	37	

a Clinicopathological variables were compared between groups with negative STC2 expression (n=94) and positive STC2 expression (n=146).

STC, stanniocalcin 2; AFP, α-fetoprotein.

**Table II:** Univariate and multivariate analysis of overall survival in 240 hepatocellular carcinoma patients.

	Univariate analysis			Multivariate analysis		
		
Variables	HR	95% CI	P-value	HR	95% CI	P-value
STC2	3.01	1.29–6.75	<0.001	2.39	1.04–5.89	0.013
Gender	0.65	0.28–1.52	0.33	-	-	-
Age	0.81	0.48–1.37	0.44	-	-	-
Tumor size	1.19	0.73–2.23	0.51	-	-	-
Histology	1.20	0.66–1.56	0.061	-	-	-
Cirrhosis	0.78	0.52–1.11	0.22	-	-	-
HBsAg	1.32	0.42–2.27	0.74	-	-	-
Serum AFP	1.59	0.92–2.74	0.09	-	-	-
Metastasis	1.49	1.13–2.43	0.019	1.21	0.88–2.93	0.035
Recurrence	1.60	1.06–2.56	0.011	1.33	0.88–3.50	0.020

HR, hazard ratio; CI, confidence interval; AFP, α-fetoprotein.
